# Microglial Activation in Metal Neurotoxicity: Impact in Neurodegenerative Diseases

**DOI:** 10.1155/2023/7389508

**Published:** 2023-01-31

**Authors:** María I. Martínez-Hernández, Leonor C. Acosta-Saavedra, Luisa C. Hernández-Kelly, Jaqueline Loaeza-Loaeza, Arturo Ortega

**Affiliations:** Departamento de Toxicología, Centro de Investigación y de Estudios Avanzados del Instituto Politécnico Nacional, Mexico City 07360, Mexico

## Abstract

Neurodegenerative processes encompass a large variety of diseases with different pathological patterns and clinical features, such as Alzheimer's and Parkinson's diseases. Exposure to metals has been hypothesized to increase oxidative stress in brain cells leading to cell death and neurodegeneration. Neurotoxicity of metals has been demonstrated by several *in vitro* and *in vivo* experimental studies, and most probably, each metal has its specific pathway to trigger cell death. As a result, exposure to essential metals, such as manganese, iron, copper, zinc, and cobalt, and nonessential metals, including lead, aluminum, and cadmium, perturbs metal homeostasis at the cellular and organism levels leading to neurodegeneration. In this contribution, a comprehensive review of the molecular mechanisms by which metals affect microglia physiology and signaling properties is presented. Furthermore, studies that validate the disruption of microglia activation pathways as an essential mechanism of metal toxicity that can contribute to neurodegenerative disease are also presented and discussed.

## 1. Introduction

Microglial cells are present in the central nervous system (CNS) within the brain parenchyma. Microglia are considered the brain “macrophages” since these cells are involved in multiple functions from the embryonic stage to adulthood, such as immune vigilance, synaptic pruning, neurogenesis, and cleansing; they also act as sensors of environmental molecules, such as ions, neurotransmitters, cytokines, chemokines, and growth factors [1–3].

Microglia are dynamic and heterogenous, and these cells can activate and change their phenotype depending on the brain microenvironment. The cells of this lineage can polarize to an “M1” or “M2” phenotype; the first one is characterized by the secretion of proinflammatory molecules such as tumor necrosis factor alpha (TNF-*α*), interferon gamma (IFN-*γ*), interleukin 1 beta (IL-1*β*), interleukin 6 (IL-6), interleukin 12 (IL-12), interleukin 23 (IL-23), nitric oxide (NO), and reactive oxygen species (ROS), while the latter phenotype secretes anti-inflammatory molecules such as interleukin 4 (IL-4), interleukin 10 (IL-10), interleukin 13 (IL-13), and arginase 1 (Arg-1) [1, 3–5]. MicroRNAs (miRNAs) play a crucial role in CNS diseases through posttranscriptional regulation. In this sense, miRNAs are essential regulators mediating microglial activation and polarization [6].

In the brain, metals play an essential role in health and disease. Metals are natural components of the earth crust disseminated to the biosphere through human activities [7, 8]. Some metals are physiologically essential, for example, cobalt (Co), chromium (Cr), copper (Cu), iron (Fe), manganese (Mn), molybdenum (Mo), nickel (Ni), selenium (Se), and zinc (Zn) among others, but can be toxic in large quantities or certain forms [9, 10]. Metals are usually essential components in biological molecules and involve multiple enzymatic reactions [11]. The difference between the deficit, physiological, and toxic metal concentrations are relatively small; therefore, it is important to have strict control of their concentrations. It is also pertinent to mention that small amounts of nonessential metals such as aluminum (Al), cadmium (Cd), mercury (Hg), and lead (Pb) can also promote severe damage since these metals disrupt the physiological activity of the essential metals [9, 10].

Neurodegeneration is thought to be the most common manifestation of metal toxicity. A link has been found between abnormal brain metal accumulation and various neurological disorders, such as Alzheimer's (AD) and Parkinson's (PD) diseases [12–14].

Environmental exposure to metals or dysregulation of this essential metals homeostasis contributes to microglial activation and, in turn, can trigger an inflammatory response, which depends on factors such as prolonged induction of cytokines, receptor activation, dysregulation of signaling pathways, or even the absence of sufficient anti-inflammatory mediators to reduce the response. This neuroinflammation can coincide with other mechanisms of neurotoxicity and cause alteration of the synaptic activity or neuronal death [12–15].

The present contribution is an approach to analyze our current understanding of the role that microglial activation plays under exposure to both essential and nonessential metals and how these processes contribute to the development of neurodegenerative diseases.

## 2. Microglia Cells

Microglia cells are among the most versatile cells in the brain, as these cells are involved in various critical actions for the development and homeostasis of the brain. Microglia represent 10%–15% of the nonneuronal cells in the brain and are generally known as resident immune cells that closely resemble peripheral macrophages [16]. These cells respond rapidly to stimuli, secrete a great diversity of signaling molecules, and, interestingly, can also change their phenotype.

Microglia play a key role in the shaping and fine-tuning of brain circuits in a healthy brain. Together, microglia and plasma membrane receptors respond to the internal and external cellular microenvironment, playing an essential role in CNS physiology and pathology [17]. Microglia express various plasma membrane and cytoplasmatic receptors (Figure 1), enabling them to participate in CNS physiology and pathology, as these cells respond immediately to the internal and external cellular microenvironment. Among these microglia receptors are the pattern recognition receptors (PRRs) that detect pathogens associated with molecular patterns (PAMPs), molecular patterns associated with tissue damage (DAMP), and neurotransmitter receptors (Figure 1).

The PRRs include Toll-like receptors (TLRs) such as TLR4 and TLR1/2 [18, 19]. Signaling through TLRs activates downstream signaling cascades through two major adapter proteins, myeloid differentiation primary-response protein 88 (MyD88), and domain-containing adaptor interferon-*β* (TRIF) that converge at the IkB kinase (IKKs) and the mitogen-activating kinases (MAPKs), leading to the activation of transcription factors, particularly nuclear factor kappa B (NF-*κ*B) and activator protein 1 (AP-1), to promote the expression of proinflammatory mediators [20].

The NOD-like receptors (NLRs) are cytosolic sensors containing NACHT and C-terminal leucine-rich repeat (LRR) domains. Upon activation by different stimuli, such as PAMPs or endogenous danger signals, the NLRP3 inflammasome is formed after the association of NLRP3 with the adaptor protein apoptosis-associated speck-like protein containing CARD, also known as PYCARD (ASC) and procaspase-1 [18, 21]. It has been shown that NLRP3 is expressed in microglia cells but not in astrocytes and that the stimulation with amyloid-*β* peptides activates NLRP3 and IL-1*β* secretion [22].

The type C receptors (CLRs), like the receptor encoding C-type lectin domain family 7 member A (CLEC7A), are involved in autophagy and phagocytosis processes, and amoeboid microglia are characterized by their high CLEC7A expression [23, 24]. Microglia also express receptors that help to endocytose apoptotic cells, aggregated proteins, and lipoprotein particles. These receptors include scavenger classes such as cluster of differentiation 36 (CD36) or *Platelet glycoprotein 4* and macrophage receptors with collagenous structure (MARCO). It has been found that CD36 is expressed in human fetal microglia, N9-immortalized mouse microglia, and the brain of AD patients [25, 26]. MARCO is responsible for the microglia actin cytoskeleton rearrangements, characterized by the fact that these cells appear round and are slightly adherent [27].

Low-density lipoprotein receptors (LDLRs) are also expressed in microglia. Apolipoprotein E (ApoE) is known to bind to microglial LDLR to become internalized *via* receptor-mediated endocytosis and regulate c-Jun N-terminal kinase (JNK) activation [28]. Three tyrosine kinase receptors (RTK), *Tyro 3* protein tyrosine kinase (Tyro3), Axl receptor tyrosine kinase (Axl), and MER protooncogene tyrosine kinase (Mertk) that regulate the innate immune response in dendritic cells and macrophages, mediate the engulfment of apoptotic cells by phagocytes that have been described in microglia [29, 30]. Mertk and Axl expression is prominently upregulated in the inflammatory environment and upon a cuprizone (Oxalic acid bis (cyclohexylidene hydrazide)) challenge [31–33].

Microglia cells express chemokine receptors, like the C-X3-C motif chemokine receptor 1 (CX3CR1) and the C-X4-C motif chemokine receptor 4 (CXCR4). CX3CR1 has a prominent microglia expression; it is a G-protein-coupled receptor and transduces several well-characterized signaling pathways leading to the activation of transcription factors, including NF-*κ*B and cAMP responsive element binding protein (CREB) [34, 35]. CXCR4 receptors mediate IL-6 upregulation *via* ERK, PI3k/Akt, and NF-*κ*B signaling pathways [36].

Other receptors expressed in microglia are integrin-like receptors, such as integrin subunit alpha M (CD11b) and integrin subunit alpha X (CD11c). Microglial activation is represented by an increased expression of CD11b and CD11c, and NO plays a crucial role in its expression [37, 38].

Purinergic receptors, such as P2Y12 (P2Y12R) and P2X7 (P2X7R) receptors, have also been reported in microglia. The P2Y12R is active in these cells under basal conditions, albeit negatively regulated after activation; it drives migration and phagocytosis [39], while P2X7R reduces microglial phagocytic capacity and produces mature caspase-1 by activating the inflammasome [40].

Adenosine receptors, such as A2a, promote the secretion of inflammation mediators and phagocytosis. Activation of microglial A2a receptors also induces the expression of cyclooxygenase 2 (COX2) mRNA, the synthesis of prostaglandin E2 (PGE2), and the potentiation of NO release from activated microglia [41].

Furthermore, microglia express immune receptors that regulate the amplitude and duration of their activation. These include the superfamily of immunoglobulin (Ig-SF) molecules that deliver stimulatory or inhibitory signals through both protein tyrosine kinase and protein tyrosine phosphatase pathways. Among the most studied of these molecules, it is pertinent to mention triggering receptor expressed on myeloid cells (TREM), an activating receptor that binds to phospholipids [42]. Expression of TREM2 is abundant in all forebrain regions. It is involved in homeostatic microglial function [43]. The sialic acid binding immunoglobulin-like lectin 3 (CD33) binds to sialic acid and triggers inhibitory signals in human microglia [44]. Low CD33 levels have been reported in newborn and adult mice; interestingly, microglial polarization with granulocyte macrophage colony-stimulating factor (GM-CSF) followed by interferon gamma (IFN-*γ*) and *Lipopolysaccharide* (LPS) has also been found [45].

CD200 is a transmembrane glycoprotein, mainly expressed in neurons that binds to its specific receptor (CD200R), expressed exclusively in microglia and macrophages [46]. The interaction CD200/CD200R maintains microglia in a quiescent state; therefore, CD200/CD200R signaling disruption can cause microglial over reactivity [47].

Interestingly, signal regulatory protein *α* (SIPR*α*; also known as SHPS-1, p84, and BIT) is a membrane protein that binds to CD47, activating the protein tyrosine phosphatases SHP-1 or SHP-2 through their cytoplasmic region [48, 49]. SIPR*α* downregulation triggers an inflammatory response in microglia, revealing an inhibitory effect of SIPR*α* in microglial activation [50].

### 2.1. Receptors for Neurotransmitters and Neuropeptides

Microglia also express multiple neurotransmitters and neuropeptide receptors involved in glial-neuronal interactions (see Figure 1) [51, 52]. These receptors allow microglia to monitor neuronal activity, supporting microglial involvement in synaptic plasticity modulation and the subsequent change in the dendritic tree density. Neurotransmitter receptors are of utmost importance since these proteins detect and eliminate damaged neurons and promote the secretion of neurotrophic factors needed for neuronal regeneration. These receptors regulate the release of inflammatory cytokines in response to several stimuli. Microglia express ionotropic and metabotropic glutamate receptors (GRI, GRM). The former are *α*-amino-3-hydroxy-5-methyl-4-isoxazole propionic acid (AMPA, GRIA), N-methyl-D-aspartate (NMDA, GRIN), and kainate (KA, GRIK) receptors [53]. Metabotropic glutamate receptors are classified according to their receptor-coupled second messenger system and their specificity for different agonists into three groups; group I includes mGluR1/5 (GRM1/5), group II includes mGluR2/3 (GRM2/3), and group III has mGluR6/8 (GRM6/8) [53].

In line with these findings, a study by Noda demonstrated that the expression of functional GRIA receptors in rat microglia might mediate neuron/microglia communication in the physiological and pathological states [54]. A study by Hagino et al. showed that the potentiation of microglial GRIA receptors serves as a negative feedback mechanism for regulating TNF-*α* release [55]. Interestingly, Fontain et al. has demonstrated an endogenous ionotropic glutamatergic transmission mediated mainly through GRIA and GRIK receptors and, to a smaller extent, by GRIN receptors, positively regulating the microglial dendritic structure and process dynamism [56]. Accordingly, Liu et al. showed that microglia exposed to glutamate increase their migration, and this chemotaxis is mediated by GRIA and GRM receptors [57].

There is also evidence supporting the microglial expression of GRIN receptors. For example, microglia are transiently activated following injections of NMDA into the cortex, and these receptors may enhance the release of TNF-*α*, IL-1, and NO [58, 59]. The stimulation of microglial GRM3 receptors prevents mitochondrial stress and apoptosis [60]. Furthermore, Taylor et al. demonstrated that stimulation of GRM2 induces TNF-*α* release, which contributes to microglial neurotoxicity *via* neuronal TNF receptor 1 and caspase-3 activation [61]. Byrnes et al. demonstrated that GRM5 receptor stimulation inhibits microglial activation *in vitro*, proliferation, NO, TNF-*α*, and ROS production [62]. More recently, Zhang et al. reported that activation of GRM5 inhibits inflammatory signaling triggered by alpha-synuclein (*α*-Syn); GRM5-mediated signaling partially inhibited microglia activation [63].

GABA is the major inhibitory neurotransmitter in the CNS, maintaining the healthy balance between excitation and inhibition in the brain, whose imbalance is significantly affected in epilepsy, AD, autism spectrum, and schizophrenia [64–66].

Gamma-aminobutyric acid (GABA) receptors are expressed in microglia. It was demonstrated that activation of GABA_B_ receptors attenuates the LPS-induced IL-6 and interleukin 12p40 (IL-12p40) release [67]. Moreover, the expression of dopamine receptors (DR) such as D1R, D2R, D3R, D4R, and D5R in microglia has been documented. Also, it was observed that in a damaged brain, the expression of D2R is present in ionized calcium-binding adapter molecule 1 (Iba-1) immunoreactive inflammatory cells (microglia) [68].

Microglia express and respond to the muscarinic acetylcholine receptor (mAChRs) agonists. In this context, it has been observed that carbachol increases the chemotaxis activity and decreases the phagocytic activity of cultured microglia [69]. Besides, receptors for neuropeptides, such as the neurokinin-1 receptor (NK1R), are necessary for substance P- (SP-) mediated chemotaxis [70]. In this sense, the activation of bradykinin receptors, specifically the B2 and B1 receptors, amplifies inflammation mediators (TNF-*α* and NO synthesis) [52, 71]. The receptors described above are of utmost importance since their activation in microglia determines the balance between a proinflammatory or anti-inflammatory phenotype.

## 3. Microglial Activation: M1 and M2 Phenotypes

Microglia activation or polarization is often classified as classical (M1) or alternative (M2) [72], following the paradigm of macrophages [73]. In Figure 2, both microglial phenotypes are represented. M1 activation is characterized by the simultaneous activation of TLR and IFN-*γ* signaling pathway and the production of proinflammatory cytokines and chemokines, such as TNF-*α*, IL-6, IL-12, and C-C motif chemokine ligand 2 (CCL2). Moreover, NADPH oxidase generates superoxide anion and ROS, as well as inducible nitric oxidase synthase (iNOS), which converts L-arginine to NO. Another inflammatory mediator produced by M1 is matrix metalloproteinase 12 (MMP12). M1 microglia also express high amounts of major type II histocompatibility complex (MHC type II), costimulatory molecules, Fc receptors, and integrins [74].

Microglia M2 secretes growth factors such as IGF-I, fibroblast growth factor (FGF), and colony-stimulating factor 1 (CSF1), as well as neurotrophic factors like nerve growth factor (NGF), neurotrophic factor derived from the brain (BDNF), neurotrophins (NTs), and glial cell derived neurotrophic factor (GDNF). M2 activation leads to anti-inflammatory, healing, and repair activities of microglia. IL-4 can induce IL-13 and IL-10 release as well as activation of the receptor activated by the gamma peroxisome proliferator (PPAR*γ*), liver receptor X (LXR), and retinoic acid receptor (RXR), respectively [18]. Likewise, M2 activation promotes the release of anti-inflammatory cytokines, such as IL-10 and TGF-*β*, and induces Arg-1, which supports the conversion of arginine to polyamines (Figure 2). Neurotrophic factors activate tyrosine kinase receptors (RTK), which regulate synaptic strength and plasticity [4, 75].

The polarization toward M1 or M2 microglial phenotype is also regulated by miRNAs, which are molecules of 18–25 nucleotides long that regulate gene expression at the posttranscriptional level [76]. miRNAs activate microglia during inflammation [77]. The group of proinflammatory miRNAs, such as miRNA-155, is induced by LPS [78]. miRNA-155 promotes apoptosis and increases the release of proinflammatory cytokines. Another miRNA involved in the inflammatory response is miRNA-125, which is induced by TLR agonists and modulates the classical NF-*κ*B inflammatory pathway [79]. Another study identified that miRNA-101 regulates proinflammatory cytokine expression, increasing the production of IL-6 and TNF-*α* and inhibiting MAPK phosphatase-1 (MKP-1) [80].

Other miRNAs are also involved in inflammation. For example, miRNA-146 is expressed at the highest microglia levels and upregulated in all lesion types [81]. In this sense, it has been reported that during microglia activation, miRNA-21 downregulation increases the production of the Fas ligand (FasL), which mediates neurotoxicity in rat microglia [82].

It has also been observed that microglia cultured with GM-CSF and IFN-*γ* downregulate miRNA-124; these cells show an activated phenotype with a low level of miRNA-124 expression [83]. This miRNA has been considered anti-inflammatory, a two-day with miRNA-124 after an ischemic insult increases of Iba-1+ cells expressing the M2 marker CD206 and a parallel pronounced decrease of the M1 marker CD16/32; these data confirm the protective role of miRNA-124 [84].

Another miRNA expressed during the microglial activation process is miRNA-204. A study by Li et al. found that miRNA-204 inhibits the expression of Sirtuin1 (SIRT; a NAD+-dependent class III histone deacetylase) and upregulates the expression of matrix metallopeptidase 9 (MMP9), iNOS, and IL-1*β* [85]. In another study by Yao et al., it was demonstrated that miRNA-9 downregulates monocyte chemotactic protein-induced protein 1 (MCPIP1) expression and induces microglia activation [86]. A study by Kumar et al. has shown that overexpression of miRNA-26a significantly decreases the production of inflammatory cytokines such as TNF-*α* and IL-6. In contrast, the knockdown of miRNA-26a increases the expression of these mediators [87].

Interestingly, transcriptome studies show that microglial activation is varied and context-dependent. During normal CNS function, microglia are in a so-called homeostatic state in which their transcriptomic profile reflects a surveillance activity [75, 88–92]. In sharp contrast, in neurodegeneration models, microglia express neurotoxic and neuroprotective factors; genes involved in oxidative phosphorylation; lysosome, ribosome factors, miRNAs, and responses involved in misfolded proteins, stress and neuronal injury, or death [91, 93].

## 4. Microglial Activation by Essential and Nonessential Metals: Cell Mechanism and Signaling Pathways

Various studies have shown that both essential and nonessential metals can accumulate in the brain and promote microglial activation; this occurs *via* multiple receptors and signaling pathways (Figures 3 and 4).

### 4.1. Essential Metals

#### 4.1.1. Manganese (Mn)

Manganese (Mn) is a trace element essential for human and brain development. Excess manganese is neurotoxic and has been associated with neurodegenerative disorders associated with basal ganglia dysfunction, like PD and Huntington's disease (HD) [81, 94, 95]. Neurotoxicity induced by overexposure to Mn includes impaired mitochondrial function, metabolism of neurotransmitters, iron homeostasis, and induction of oxidative stress [96–99]. It has been shown to affect microglia and astrocytes, regulating the activation of proinflammatory responses, which contribute to its toxic effects [100]. *In vitro* studies have attempted to explain the molecular mechanism by which Mn has its neurotoxic effects. A report by Filipov et al. [101] describes that Mn moderately increases IL-6 and TNF-*α* production at cytotoxic concentrations. Moreover, Zhang et al. using a HAPI microglia cell line and exposure to 10 *μ*M manganese chloride (MnCl_2_) for 2 h reported an increased ERK and p38 activation [102]. Furthermore, Crittenden and Filipov demonstrated that p38 is critical for the Mn-induced potentiation of cytokine production to occur [103]. In the same line, a Kirkley et al. study showed that treatment with Mn in primary microglia cultures led to an increase in the proinflammatory gene expression of nitric oxide synthase 2 (Nos2), IL-1*β*, and caspase 1, resulting in the transition to a mixed M1/M2 phenotype and a debranched morphology [104]. Wang demonstrated that Mn activates the NLRP3-CASP1 inflammasome pathway in mice hippocampus and BV2 cells by triggering autophagy-lysosomal dysfunction. In a study carried out by Popichak et al. in which a mixed glial culture (astrocytes and microglia) was used, an MnCl_2_ exposure increased the inflammatory genes Nos2, TNF-*α*, Cc15, IL-6, Ccr2, and IL-1*β* expression (see Table 1) [105]. One study by Chen et al. showed that Mn exposure induced autophagy dysfunction *in vivo* and *in vitro* and confirmed the role of leucine-rich repeat kinase 2 (LRRK2) in Mn-induced microglia neuroinflammation [106]. A report by Sarkar et al. demonstrated an increase in NLRP3 and maturation of the inflammatory cytokine IL-1*β* [107]. The relevant information of Harischa et al. showed that microglia exposed to Mn stimulated the release of *α*-Syn-containing exosomes and exhibited a pronounced amoeboid morphology resulting from the activation and formation of blebs and filopodia, like those present in other phagocytic cells. Also, the expression of Iba-1 and iNOS and the release of proinflammatory cytokines (IL-12, IL-1b, and IL-6) were significantly increased [108]. Ultimately, a study by Lin et al. reported that Mn alone did not affect amyloid-beta precursor protein (APP) and *β*-secretase (BACE1) expression and A*β* generation in N2a cells unless the cells were cocultured with microglia or microglia conditioned medium, pointing out that Mn treatment increased the expression level of APP, BACE1, amyloidogenic C99 fragment, and A*β* [109] (see Table 1 and Figure 3).

#### 4.1.2. Iron (Fe)

Iron (Fe) is involved in many brain cellular processes: respiration, myelin synthesis, DNA synthesis, oxygen transport, metabolism of neurotransmitters, and many others [110]. Excessive Fe deposition has been reported in the CNS in several neurodegenerative pathologies such as AD, PD, HD, and amyotrophic lateral sclerosis (ALS) [111]. Fe is present in neurons, oligodendrocytes, astrocytes, and microglia. Within the cell, Fe mediates essential functions due to the ability to participate in electron transfer reactions, switching between two states: ferrous (II) and ferric (III) Fe. This mechanism represents a double-edged sword since the different levels of ROS are produced in these reactions allowing calcium-mediated basal synaptic transmission and the release of proinflammatory cytokines, thus creating a proinflammatory environment [112, 113].

Microglia is capable of being more efficient in Fe sequestration compared to the other brain cells. In the study by Healy et al., it is reported that ferritin is expressed in oligodendrocytes and microglia; therefore, iron accumulation loading with ferrocene affects glial morphology and number. A significant 15% increase in the number of Iba1-positive microglia was observed [114]. In another study, Bishop observed that microglia were the most efficient brain cell in accumulating Fe, followed by astrocytes and neurons [115]. On the other hand, the study by Yauger et al. demonstrated that exposure to Fe in primary microglia cultures increased ROS levels [116]. These studies documented that an increase of Fe in microglia cells led to the deregulation of iron homeostasis, either due to its excessive accumulation or modification in iron transporters. In another study by Rathore et al., the authors demonstrate that TGF-*β*1 and TNF-*α* combined with Fe reduce Fe reduce (FPN) mRNA levels and increases H-ferritin mRNA [117]. These results suggest that both cytokines promote iron uptake and retention in microglia. A study by Zhang et al. showed that exposure to Fe leads to microglial activation and enhances neurotoxicity [118]. These results demonstrate that activated microglia produce a large amount of reactive oxygen species (iROS) and a morphological alteration. The increase in mRNA and protein levels of PKC-*δ*, P38, ERK1/2, JNK, and NF-*κ*B (p65) was also observed (see Table 1 and Figure 3).

#### 4.1.3. Copper (Cu)

Copper (Cu) is a metal needed for the function of many enzymes. It functions as a cofactor and structural component of several enzymes; therefore, copper participates in many physiological pathways, including energy metabolism, antioxidative defense, and iron metabolism [119]. Alterations in brain Cu homeostasis have been implicated in AD and PD [119–123]. Although the precise mechanisms by which oligomeric A*β* species exert their toxic effects are unknown, Cu may exacerbate the toxicity of A*β* oligomers through the formation of ROS, as A*β* can mediate the reduction of Cu^2+^ to Cu^+^ [124].

A study by Hu et al. demonstrated that in microglia cells, Cu exposure increases TNF-*α*, NO, and iNOS levels [125]. It was found that both BAY11-7082 and SC-514, inhibitors of I*κ*B-*α* phosphorylation and IKK-2, respectively, block Cu (II)-induced TNF-*α* or nitric oxide release in BV2 cells, suggesting a role of NF-*κ*B in Cu (II) actions. Moreover, Cu can trigger an inflammatory process; in a study by Yu et al., it was observed that Cu (II) combined with beta-amyloid protein (A*β*) induced a phenotype of activated microglia, and the release of cytokines such as TNF-*α* and NO, the increase in NO, was accompanied by the expression of iNOS [126]. Kitazawa et al. found that a 24 h Cu exposure inhibits the phagocytic activation of the BV2 microglia cell line with an increase in proinflammatory cytokines such as IL-1*β*, TNF-*α*, and IL-6 release [127] (see Table 1 and Figure 3).

#### 4.1.4. Zinc (Zn)

Zinc (Zn) is one most abundant trace elements in the brain, and it is involved in multiple functions. Zn regulates gene expression through transcription factors activity; it is responsible for the action of enzymes in metabolism and modulates various signaling pathways [128, 129]. Disruption of Zn homeostasis has been linked to neurological abnormalities, including depression, schizophrenia, AD, PD, and ALS [130]. Furthermore, released Zn by neurons under several conditions causes microglial activation and the release of proinflammatory cytokines that could cause damage to the myelin sheaths [131].

A study by Kauppinen et al. showed that Zn directly triggers microglial activation and increases NF-*κ*B and NO production, and the glycoprotein F4/80 expression was also increased [133]. Extracellular Zn triggers microglial activation by activating NADPH oxidase, PARP-1, and NF-*κ*B. Moreover, Higashi et al. demonstrated that Zn facilitates the expression of iNOS mRNA [134] (see Table 1 and Figure 3).

#### 4.1.5. Cobalt (Co)

Cobalt (Co) is an element present in the earth's crust; it is essential for mammals in the form of cobalamin (vitamin B12). The sources of Co in the air are both natural (volcano eruptions, erosion, and forest fires) and anthropogenic (burning of fossil fuels, engine emissions, and disposal of alloys) [138]. Available data on the toxic effects of Co include DNA fragmentation, caspase activation, increased ROS production, and MAPKs phosphorylation [139–142].

Excess Co is cytotoxic and neurotoxic, a study carried out by Mou et al. showed that in the N9 microglia cell line, exposure to Co induces NO production, cytokines (TNF-*α* and IL-6), and chemokine synthesis, in addition to the regulation of iNOS mRNA [135]. The production of Co-induced cytokines involves NF-*κ*B as well as p38 MAPK signaling and ROS participation in microglial activation, suggesting that Co neurotoxicity should also be attributed to microglial activation that could potentiate neuronal injury through the increase of proinflammatory mediators. Another study by Kim et al. showed that CoCl_2_ induces hypoxia factor 1 (HIF-1) expression, inhibits the inflammasome NLRP3, and attenuates the release of caspase 1 and IL-1*β* [136]. In another study by Merlo, CoCl_2_ was shown to induce HIF-1 and NF-*κ*B in rat microglial culture [137] (see Table 1 and Figure 3).

### 4.2. Nonessential Metals

#### 4.2.1. Lead (Pb)

Lead (Pb) is a heavy metal widely distributed in the environment, and overexposure to this metal can affect CNS function, especially learning and memory [143, 144]. Some individuals chronically exposed to Pb have been diagnosed with learning disabilities and have difficulties in listening, speaking, reading, writing, reasoning, or mathematical abilities [145]. Disability from Pb overexposure is primarily related to neuronal injury or death [146]. Some studies have indicated that Pb can interfere with calcium signaling, suppress neurogenesis and neuronal differentiation, influence neurotransmitter release, and increase the production of A*β* [147–149]. Exposure to Pb in microglial cells results in their activation and morphological change, as well as in the induction of proinflammatory cytokines [150, 151].

*In vitro*, Pb exposure significantly increases microglial activation and upregulates TNF-*α*, IL-1*β*, and iNOS release [148]. A study by Liu et al. demonstrated that Pb exposure could induce significant microgliosis in the hippocampus of young mice, which is mediated most possibly through the activation of the TLR4/MyD88/NF-*κ*B signaling cascade, augmenting the expression of inflammatory the cytokine IL-1*β* and TNF-*α* and the activation of p38-MAPK and ERK1/2 [152]. Flores-Montoya et al. showed that a low Pb concentration exposure decreases C-C chemokine receptor type 7 (CCR7) mRNA levels in microglia cells, whereas a high Pb concentration exposure diminishes MHCII levels [153]. Mu et al. reports that exposure to Pb^2+^ increases ROS and TNF-*α* levels and significantly impacts the expression of 16 genes related to oxidative stress and antioxidant defenses in microglia BV-2 cells [154] (see Table 2 and Figure 4).

#### 4.2.2. Aluminum (Al)

Aluminum (Al) is a ubiquitous metal in the environment and is often used in industry to make kitchen utensils and as a pharmacological agent (antacids and antiperspirants). It is bioaccumulated after prolonged use or exposure [155]. Al exposure influences several significant reactions that result in various effects on the CNS. It affects axonal transport, neurotransmitter synthesis, synaptic transmission, protein phosphorylation/dephosphorylation, protein degradation, and inflammatory response gene expression [156]. Al^3+^ can bind strongly to metal-binding amino acids (histidine, tyrosine, arginine, etc.) or phosphorylated amino acids, resulting in protein oligomerization and inducing conformational changes that inhibit its degradation by proteases [151, 152]. By exhibiting single oxidation, Al^3+^ also binds to nucleoside phosphate groups, such as adenosine triphosphate (ATP). Therefore, it can influence energy metabolism. Al has been linked to several neurodegenerative diseases, including AD, PD, and ALS [157–160].

A study by Akinrinade et al. showed an increase in lipid peroxidation products in the brain and ROS formation after Al exposure [161]. Furthermore, an inflammatory response is also activated, increasing astrocytic and microglial activation (see Table 2 and Figure 4).

#### 4.2.3. Cadmium (Cd)

Cadmium (Cd) is a ubiquitous industrial and environmental pollutant. It accumulates in humans and animals. The sources of human exposure to Cd are primarily anthropogenic activities such as the primary metals industry, production of batteries, consumption of contaminants, food and water, tobacco smoke, and polluted air [162]. Cd also reaches the CNS, causing neurological alterations and leading to memory and attention dysfunctions [162]. The cellular and molecular basis of Cd neurotoxicity are not precise; however, in a diversity of models of neuronal and glial cells exposed to Cd, an increase in ROS production, cell death, and disturbance of cell signaling pathways are present [162–164].

Yang et al. [165] demonstrated that in primary microglia cultures, Cd induces microglial activation through the production of ROS and the activation of transcription factors sensitive to redox, like NF-*κ*B and AP-1, which leads to the expression of genes related to oxidative stress. Another study *in vivo* and *in vitro* by Khan et al. [166] showed that in the microglial cell line, BV-2 increased the levels of p-NF-*κ*B. In the brain cortex and hippocampus, an augmentation of the microglia marker Iba-1 was reported, as well as an increase in TNF-*α*, IL-1*β*, NOS2, ROS, lipidic peroxidation (LPO), p-NF-*κ*B, Bax, caspase 3, and PARP-1 (see Table 2 and Figure 4).

## 5. Metal Toxicity as a Risk Factor for Neurodegenerative Diseases

Neurodegenerative diseases, including AD and PD, have attracted attention in recent decades due to their high incidence worldwide. The etiology of these diseases is still unclear. However, the role of the environment as a risk factor is well documented.

Homeostasis of metal ions plays a vital role in health and neurodegenerative diseases by influencing cellular biochemical pathways. The alteration of some metal ions can lead to cytotoxic effects linked to neurodegenerative disorders such as AD and PD. Excessive concentration of nonsequestered metals can cause toxicity. In addition to altering the membrane potential, metal ions can bind to and affect protein/enzyme and nucleic acid activity, particularly in neurons. Furthermore, the leading cause of transition metals' oxidative toxicity is ROS generation, the most penetrating oxidant in cells [99, 111, 119, 123, 130].

The exact mechanism by which metals induce toxicity is not fully understood, and each metal could likely be toxic through specific pathways. Of particular importance, oxidative stress and neurodegeneration have been reported as consequences of toxic exposures to essential and nonessential metals, along with dyshomeostasis in primary metal metabolism [167].

There is evidence of the effects of metals and their relationship with neurodegenerative diseases, as well as reports on the presence of metals in the brain of patients with AD and PD, as will be described below.

### 5.1. Alzheimer's Disease (AD)

AD is the most common disease of aging and is usually considered a cognitive disorder. One of the most common neuropathological hallmarks of AD is the misfolding and aggregation of the *β*-amyloid peptides, senile plaques, or amyloid plaques, which mainly consist of small *β*-amyloid peptide (A*β*) (up to 42 or 43 amino acids long) [168, 169].

Several studies demonstrate the relationship between exposure to Mn and AD. In the study by Tong et al., a significant correlation of Mn with the Mini-Mental State Examination score and Clinical Dementia Rating Scale score was found. In addition, plasma A*β* peptides increased with elevated Mn concentrations [170]. Fe is another metal that contributes to the deposition of A*β* and the formation of neurofibrillary tangles, which promotes AD development. Brain Fe and A*β* plaques colocalization was confirmed with a quantitative susceptibility map (QSM) [171]. An analysis of AD human brains showed increased levels of Cu and Zn compared to control brains; this fact validates the hypothesis that the change in metal speciation due to the accumulation of A*β* and tau affects the brain metals homeostasis [172]. A recent meta-analysis suggested that a slight increase in serum Cu may represent a risk factor for AD [173]. In a study by Lovell et al., Zn levels are increased in senile plaque derived from patients diagnosed with AD [123]. The correlation between Co and AD or other neurodegenerative diseases is not clear. However, common mechanisms of neurotoxicity might be present. In one clinic report of a patient with arthroprosthetic cobaltism and sural nerve biopsy, neurotoxicity occurs through demyelination and axonal loss [174]. Another study by Bridges et al. demonstrated that all scanned patients had regions of significant hypometabolism and neurological toxicity from elevated systemic cobalt [175] (see Table 3).

In patients with AD, Pb levels were found to be significantly higher respect to normal subjects [176]. In the same line, increased Al levels have been traditionally linked to the pathogenesis of AD due to its accumulation in the brain [177]. Some reports have demonstrated, using histopathology, the presence of Al and amyloid plaques in different brain regions, as well as the presence of Al in glial cells [178–181]. A recent study by Exley and Clarkson confirmed that the Al content of brain tissue in AD, autism spectrum disorder, and multiple sclerosis (MS) is significantly elevated [182]. Furthermore, another study demonstrated that Al is considerably higher in MS than in non-MS [183]. Cd may also induce neurotoxicity by changing the permeability of the blood-brain barrier and interacting with other neurotoxicants, leading to A*β* aggregation and tau neurofibrillary tangle production [162]. One study using *post-mortem* brain tissue found that the AD brain had a higher concentration of Cd in the hippocampus and cerebral cortex [184]. Moreover, in a recent study using *post-mortem* brain samples from AD patients and controls, Cd concentration on the frontal cortex was lower in AD cases than in control [185]. In a meta-analysis, it was found that circulating Cd concentrations (blood, serum, or plasma) were significantly higher in AD [186] (see Table 3).

### 5.2. Parkinson's Disease (PD)

PD is a complex neurodegenerative disorder with motor and nonmotor symptoms due to a spreading process of neuronal loss in the brain. A hallmark of the disease is an aggregation of the protein *α*-synuclein (*α*-Syn), which is toxic to neurons [187].

Mn is an essential mineral, but chronic exposure to high concentrations, such as it is experienced by welders, is associated with PD symptoms. On the other hand, exposure to Mn has been suggested as a PD environmental risk factor. However, *manganism* does not involve degeneration of the nigrostriatal dopaminergic system as in PD [189, 190]. Fe has long been described to be involved in the pathogenesis of PD. It has been observed that levels of Fe, both in its ferrous (Fe^2+^) and ferric (Fe^3+^) forms, are present in Lewy bodies (LB), as well as in many other amyloid structures [191–193]. A study by Chen et al. [194] demonstrated increased iron levels in the *substantia nigra* in PD patients.

Rose et al. demonstrated that Cu (II) ions accelerate the aggregation of *α*-Syn into fibrillar plaques, the precursors to LB [195]. However, other studies showed that in PD patients, the blood concentration of copper, ceruloplasmin, its oxidase activity, and the copper atoms per ceruloplasmin molecule were lower than in age-matched healthy individuals [196, 197]. Specifically, in PD, numerous lines of evidence indicate that aberrant Zn metabolism plays a role in the neurodegenerative cascade. The study of Kumar showed that rats treated with Zn for up to 8 weeks presented decreased locomotor activity, reflecting reduced dopamine in tyrosine hydroxylase positive cells and alteration in multiple antioxidant systems [198] (see Table 4). One meta-analysis by Du et al. suggests that reduced Zn levels in the serum and plasma are associated with an increased risk for PD [199]. Another study by Dos Santos et al. showed that patients with depression and patients with one or more of the psychotic complications of hallucination, illusion, paranoid ideation, altered dream phenomenon, and confusion exhibited significantly higher Zn concentrations in hair [200]. Another study demonstrated that plasma selenium (Se) and Fe concentrations were increased considerably, whereas Cu and Zn concentrations decreased in PD patients compared to controls [201].

Although the role of Co in PD pathogenesis has not been well documented, several reports suggested that CoCl_2_, as hypoxia mimetic, can induce oxidative stress in cultured neuronal cells. It is reported that one of the mechanisms underlying CoCl_2_-induced neuronal damage is associated with the production of ROS [142, 202]. In one case study by Woelber et al., a serum Co level of 116 *μ*g/L was measured shortly after subthalamic deep brain stimulator (DBS) implantation in PD patients, and revision arthroplasty was performed using ceramic-on-polyethylene bearings [203]. After revision, the patient's serum cobalt level fell below 1 *μ*g/L, and the PD symptoms improved. Correlation studies between Co levels in the blood or brain tissue *post-mortem* are few or nonexistent. However, a recent study by Li et al. demonstrated that blood Co is associated with alterations of the blood-brain barrier and augmented oxidative stress [204] (see Table 4).

One large case-control study reported by Weisskopf et al. documents that higher accumulative exposure to Pb is associated with an increased risk of PD [205]. Also, increased Al levels have been reported in PD patients compared to controls or patients with other diseases [206, 207]. Ahmed and Santosh found that serum Al level was significantly increased in PD patients [208]. It should be mentioned that the pathogenic processes following Cd exposure result in severe cognitive impairment and are a risk factor for AD and PD [209, 210]. Individuals with AD or PD diseases present a marked loss of *locus coeruleus* neurons in which increased Cd levels were found [211]. Another study concluded that patients developed Parkinsonian features three months after Cd exposure [212]. These results suggest that Cd intoxication may damage the basal ganglia, resulting in Parkinsonism (see Table 4).

### 5.3. Microglia miRNAs Involvement in the Neurodegenerative Diseases

In recent years, increased attention has been focused on miRNAs and their relationship to neurodegenerative diseases. Many miRNAs are expressed in the brain and found as cell-free miRNAs in body fluids [213].

In microglia cells, several miRNAs contribute to the regulation of microglial polarization. Microglia-mediated mechanisms of neurotoxicity are likely to be mediated through the release of miRNAs into the extracellular environment [6, 77, 214, 215]. Dynamic mRNA regulation of neuroinflammation in astrocytes reactivity and microglia has been observed [216]. In general, miRNA-326, miRNA-155, and miRNA-27b are believed to preferentially drive a proinflammatory response, while miRNA-223, miRNA-146a, miRNA-124, and miRNA-21 are more associated with anti-inflammatory effects and let-7 family to mixed immunomodulatory regulation [216]. It is clear that specific miRNAs are involved in the development of AD, playing a role in the regulation of A*β* deposition, Tau hyperphosphorylation, synaptic dysfunction, neuroinflammation, and autophagic dysfunction [215].

Some studies correlate the levels and regulation of specific miRNAs, the molecular mechanisms triggered in microglia, and their relationship with PD. Microglia cells have been observed to respond to IL-1*β*+A*β*42-peptide-induced stress by a significant NF-*κ*B-modulated upregulation of miRNA-125b and miRNA-146a [215]. A research report by Xing demonstrated that miRNA-206 upregulation enhanced LPS-induced inflammation and A*β* release in microglia by directly targeting the 3′-UTR of IGF1 [214].

Presenilin 2 (PSD2) is a membrane-associated protease that regulates proinflammatory microglial behavior. Its deficiency or dysfunction results in uncontrolled proinflammatory activation contributing to AD [6]. In this context, a study by Jayadev et al. found that PSD2 KO microglia express higher levels of the miRNA-146 target protein IL-1 receptor-associated kinase-1 and have increased NF-*κ*B transcriptional activity [217].

In the context of neurodegenerative diseases, a study by Yao et al. demonstrated that miRNA-124 could inhibit neuroinflammation in the development of PD by regulating the MEKK3/NF-*κ*B signaling pathways and implicated miRNA-124 as a potential therapeutic target of holding the inflammatory response in PD [218].

### 5.4. Metals Regulate miRNAs in Brain Cells

The cumulating evidence linking miRNAs to environmental chemicals, coupled with the unique regulatory role of miRNAs in gene expression, calls for a correlation between metal exposure and a differential miRNAs expression pattern [219, 220].

In this context, exposure to metals, such as Mn, releases extracellular miRNAs by altering the exosomal pathway in a PD model. A marked Mn-induced increase of miR-125b, a known proinflammatory miRNA, is present [221]. Moreover, Grogg and coworkers showed that miRNA-155 expression decreases upon Mn exposure [222]. In this sense, another study by Tarale et al. demonstrated that the expression of miRNA-7 and miRNA-433 was significantly reduced upon Mn exposure. The authors identified *α*-Syn and fibroblast growth factor 20 (FGF20) as targets of miRNA-7 and miRNA-433. The reduction in these two miRNA levels causes increases in *α*-Syn and FGF-20 [223].

In human primary microvascular cells (MVECs) and a mouse model of AD, it was observed that miRNA-200b-3p, miRNA-200c-3p, and miRNA-205-5p were significantly elevated within the 24 h exposure to Cu. These results support the critical regulatory role of these miRNAs in Cu-induced loss of lipoprotein receptor-related protein 1 (LRP1) [224].

Other miRNA studies in neuronal cells have focused on miRNA-146a. A study by Pogue et al. demonstrated that the NF-*κ*B-sensitive, miRNA-146a-mediated complement factor H gene expression might contribute to inflammatory responses in Al-stressed human neuronal cells [225]. A study by Lukiw and Pogue showed that ROS-generating Al neurotoxic metal sulfates also upregulate a specific set of miRNAs that includes miRNA-9, miRNA-125b, and miRNA-128 [226].

It has also been reported that Al downregulates TREM2 expression, an effect sensitive to NF-*κ*B and miRNA-34a. It can affect microglial phagocytic capacity and contribute to the absorption and aggregation of A*β*42, amyloidogenesis, and inflammatory degeneration of the brain [188] (see Figure 4).

## 6. Future Directions

As life expectancy increases, so has the incidence of degenerative diseases, with aging as a significant risk factor. Neurodegenerative diseases such as AD affect approximately 47 million people worldwide, while PD is the second most common neurodegenerative disorder.

In AD, features of microglia that relate to phagocytosis are beneficial, whereas those related to inflammation are detrimental. Microglia can be neuroprotective by degrading A*β* plaques. Depletion of microglia also results in increased plaque load, indicating that the newly recruited population has different phagocytic properties from intrinsic microglia. The phagocytic activity of microglia is attenuated by proinflammatory cytokines [227], suggesting that microglia committed to an inflammatory response may have a lower phagocytotic capacity. In studies with anti-inflammatory drugs, microglia suppression of the inflammatory response attenuates symptoms in a mouse model of AD.

In PD pathology, *α*-Syn is secreted to the extracellular space from neurons and detected in the extracellular biological fluids in PD patients [228]. Extracellular *α*-Syn directly activates microglia and triggers a proinflammatory phenotype [229, 230]. Ultimately, *α*-Syn-induced microglial activation promotes *α*-Syn phagocytosis *via* microglial Fc*γ*R receptor and subsequently results in a series of proinflammatory events such as NF-*κ*B (p65) nuclear translocation leading to an elevated release of cytokines, potentiating the loss of DA neurons and chronic neurodegeneration in PD [231].

Metal ions have been implicated in these and other degenerative diseases, as several proteins undergoing amyloid aggregation have been identified as metal-binding proteins, generation of ROS, and change of proteins involved in signaling pathways that control diverse cellular processes such as apoptosis, energy metabolism, cells growth, and inflammation. Prolonged exposure to a metal mix can cause alterations in microglial function, from the loss of the ability to engulf proteins to the lack of control of the inflammatory response, causing an oxidative microenvironment that leads to neuron death and neurodegeneration.

Ultimately, reactive microglia cells are likely to play a vital role in disease progression and may lead to the identification of early biomarkers. Since these cells can drive functional changes in astrocytes, oligodendrocytes, neurons, and other brain cells [232, 233], these cells represent attractive drug targets to stop or limit disease progression. Previously, biomarkers from blood, plasma, serum, and cerebrospinal fluid (CSF) have been proposed. The most used biomarkers in AD are A*β*42, total Tau, and phospho-Tau in CSF, while *α*-Syn is the most promising biomarker for PD.

Several miRNAs have been identified as ideal biomarkers; these molecules are stable and easily detectable in biofluids, including plasma, serum, CSF, and urine. Cell-free miRNAs are associated with protein complexes (like the Argonaute protein family or lipoproteins) and encapsulated in vesicles, microparticles, exosomes, or apoptotic bodies). This association with proteins and vesicles protects miRNAs from being degraded by RNases in the extracellular environment [76]. Furthermore, circulating miRNAs are stable and resistant to low and high pH levels and freeze–thaw cycles, making them ideal biomarkers for pathological conditions.

In humans, it is evident that environmental factors, including toxic metals, organic pollutants, and drugs, can influence miRNA expression and function [220]. Dysregulation of specific miRNAs can contribute to microglial hyperactivation, persistent neuroinflammation, and abnormal macrophage polarization in the brain [214].

Furthermore, miRNAs may contribute to neurodegenerative diseases in response to environmental toxicant exposure *via* increasing oxidative stress and triggering inflammatory responses. Therefore, miRNAs play a dynamic role in many biochemical pathways in the mammalian brain, including neuroplasticity, stress responses, and cellular signaling, and have become key players in the neurodegenerative phenotype of AD and PD [76].

Emerging evidence suggests that miRNAs can ameliorate degeneration by inhibiting microglial activation in the brain. Suppression of microglial activation could be a therapeutic approach to protect neurons and, thus, treat or prevent neurodegenerative diseases [234].

## 7. Conclusion

As described, neurodegenerative processes in diseases like AD, PD, and others are likely to be induced by metals. Therefore, it is essential to continue the characterization of the deleterious effects of metal ion exposure in brain cells as a preliminary step to the elucidation of the cellular and molecular mechanisms that trigger the excess or deficiency of metals, as well as the alterations that these metals cause on the different cells such as astrocytes, neurons, and microglia.

Acute and chronic exposures to an endless number of metal contaminants present in water, air, soil, food, and products of daily use must be controlled. It should be taken into consideration that the possible onset of CNS pathologies may be due to contamination *per se* since we are exposed to these agents from the early stages of neurodevelopment to the rest of our lives. For this reason, toxicological evaluation of xenobiotics *in vivo* and *in vitro* systems is of vital importance.

## Figures and Tables

**Figure 1:** Receptor repertoire in microglial cells. Microglia cells express several families of receptors. ApoER2 belongs to the low-density lipoprotein receptors and is known to bind to and internalize apoE-containing lipoproteins. Tyro3 is an RTK involved in microglial activation. CD36 is a representative type C receptor with scavenger function involved in A*β* clearance. The stimulation of P2X7R, a purinergic receptor, can increase cytoplasmic calcium levels and the enhanced superoxide anion. A2a is an adenosine receptor that induces expression of NGF, COX-2 mRNA, and synthesis of PGE2. TLR4 is a member of the pattern recognition receptors family and was shown to be essential for microglia to induce proinflammatory cytokine release and ROS production; CD47 participates in the phagocytic functions of microglia. Nod-like receptors (NRL) are a family that regulates inflammation, cell death, proliferation, and transcriptional reprogramming of immune genes. CD11B is a *β*-integrin receptor, and its expression corresponds to the severity of microglial activation. mGluR is a metabotropic receptor, and its activation induces neurotoxic microglial phenotype and TNF-*α* release; NMDAR activation in microglia leads to NO release in response to NF-*κ*B signaling. AMPAR modulates TNF-*α* release.

**Figure 2:** Microglial activation, either M1 or M2, can be triggered by intrinsic or extrinsic stimuli. Stimuli can be signals of neuronal damage, neurotransmitter release, altered ion, and metal concentrations. Microglial M1 activation increases immune stimulation, blocks axonal remodeling, and neurogenesis and triggers neuroinflammation, a phenomenon characteristic of neurodegenerative diseases, by releasing inflammatory cytokines that disrupt the neuronal network. M2 microglial activation is distinguished from M1 by neuroprotection and neuronal regeneration and tissue remodeling functions and by its releasing factors like arginase-1, IL-10, IL-4, IL-13, CD206, and TGF-*β*.

**Figure 3:** Microglia activation by essential metals. In general, it has been shown that microglial activation by excess or dysregulation of essential metals (manganese, iron, copper, zinc, and cobalt) triggers an inflammatory response. This inflammatory response results from activating PI3K, PKC, and MAPK pathways through tyrosine kinase receptors or after metal entry into the cell through metal transporters such as DMT1. This signaling triggers the nuclear translocation of transcription factor as C-Jun, HIF-1, and NF-*κ*B, which induces gene expression such as nitric oxide synthase 2 (NOS2), TNF-*α*, Ccr2, IL-6, caspase 1, Cc15, and IL-1*β*. The inflammasome formation and the release of several inflammatory proteins in extracellular space are observed. By another hand, the deregulation of essential metals increases the production of O2.-, ROS, and NO. In the microglia is also reported the influence of essential metals on glycoprotein F4/80 expression and other receptors scarcely studied. SOS: son of sevenless; PI3K: phosphatidylinositol-4-5, bisphosphate 3 kinase; PKC: protein kinase C; PKC-*δ*: protein kinase delta; RAC: rac family small GTPase; JNK: c-Jun N-terminal kinase; RAS: small GTP-binding protein; Raf: serine/threonine kinase; MEK: mitogen-activated protein kinase/ERK kinase; DMT1: divalent metal transporter 1.

**Figure 4:** Activation of microglia by nonessential metals. It has been shown that nonessential metals (lead, aluminum, and cadmium) can activate microglial cells to an M1 phenotype; this activation does so through TLRs receptors *via* MyD88 and TREM2 receptors with the subsequent downstream cascade of IRAK (family of kinases) activation. Both pathways lead to the transcriptional activation of inflammatory genes and the secretion of proinflammatory interleukins such as TNF-*α* and IL-1*β*. Another signaling pathway is started by death receptors that activate apoptotic genes. In addition, exposure to these metals can increase reactive ROS and NO and trigger apoptosome formation influenced by the Bax mitochondrial release. A novel mechanism by which Al could favor the accumulation of amyloid-beta (A*β*) protein is through the activation of NF-*κ*B and increased levels of miRNA-34a, which in turn decreases the levels of the TREM receptor that inhibits phagocytosis and thus induces the accumulation of the A*β*42 protein. The Pb deregulation in microglial cells inhibits CCR7 and MHCII receptors (TRADD (tumor necrosis factor receptor-associated DEATH domain protein); FADD (Fas-associated protein with death domain); Syk (tyrosine-protein kinase); DAP12 (transmembrane adapter well known for its role in transducing activation signals); tBID (truncated p15 BID (BH3-domain-only pro-apoptotic member)); Bax (Bcl-2 associated x-protein); and P (phosphorylation)).

**Table 1:** Effects in microglia cells by essential metal.

Metal	Model	Time exposure	Concentration	Findings	Ref.
Manganese (Mn)	N9 murine microglial cell line	24 h	50-1000 *μ*M MnCl_2_	↑ IL-6 and TNF-*α* production only at higher [MnCl_2_]	[101]
	HAPI rat microglia cell line. Primary microglia culture (SD rats)	0.25, 1, 3, 6, or 24 h	0.33, 1, 3.33, 10, or 3 *μ*M MnCl_2_	↑ ERK and p38 activation in 10 *μ*M of MnCl_2_ in 2 h	[102]
	N9 murine microglial cell line	15 min, 1, 3, 4 h	250 *μ*M MnCl_2_	↑ p38 is critical for the Mn-induced potentiation of cytokine production.	[103]
	Primary microglia culture, C57BL6/J mouse	24 h	0, 10, 30, or 100 *μ*M MnCl_2_	↑ Gene expression of NOS2, TNF-*α*, IL-1*β*, IL-6, and caspase 1. ↑ Transition to a mixed M1/M2 phenotype and debranched morphology	[104]
	BV2 cell line	6 h	100 *μ*M MnCl_2_	↑ NLRP3-CASP1 inflammasome pathway	[132]
	Primary microglia culture, C57BL6/J mouse	24 h	0-100 *μ*M MnCl_2_	↑ Expression of inflammatory genes NOS2, TNF-*α*, Cc15, IL-6, Ccr2, IL-1*β*	[105]
	BV2 cell line	24 h	30 *μ*M MnCl_2_	↑ Autophagy dysfunction; role of LRRK2	[106]
	Primary microglia culture, C57BL6/J mouse ASC-CFP microglial cell line	3, 6, or 24 h	100 *μ*M MnCl_2_	↑ NLRP3 and maturation of the inflammatory cytokine IL-1*β*	[107]
	Primary microglia cultures, C57BL6/J mouse	24 h	300 *μ*M MnCl_2_	↑ Expression of Iba-1 and iNOS ↑ IL-12, IL-1*β*, and IL-6	[108]
	BV2 cell line	24 h	0, 100, and 500 *μ*M MnCl_2_	↑ The expression level of APP, BACE1, amyloidogenic C99 fragment, and A*β*. ↑ IL-1*β* and TNF-*α*	[109]

Iron (Fe)	Primary microglia culture (SD rats)	24 h 30 min	5, 25, and 100 *μ*M FeCl_2_	↑ Production O2^•-^ and iROS, ↑morphological alteration. ↑ mRNA and protein levels of PKC-*δ*, P38, ERK1/2, JNK, and NF-*κ*B (p65)	[118]
	BV2 cell line Primary microglia culture (SD rats)	24 h	100 *μ*M FeSO_4_	↑ Levels of ROS	[116]
	Organotypic hippocampal culture (SD rats)	12 h	1 *μ*M ferrocene C_10_H_10_Fe	↑ 15% in the number of Iba1-positive microglia	[114]
	Primary microglia culture, C57BL6/J mouse	6 or 24 h	20 *μ*M FeCl_3_ and cytokine TNF-*α* (10 ng/mL) or TGF-*β*1 (5 ng/mL	TGF-*β*1 and TNF-*α* induce ↓ FPN mRNA levels at 24 h ↑ H-ferritin mRNA at 6 h in microglia	[117]
	Primary microglia culture, C57BL6/J mouse	24 h	100 *μ*M ferric ammonium citrate, C_6_H_8_FeNO_7_	↑ Accumulation of iron	[115]

Copper (Cu)	BV2 cell line Primary microglia culture (SD rats)	12 h	20 *μ*M CuCl_2_	↑ Levels of TNF-*α*, NO, and iNOS	[125]
	BV2 cell line Primary microglia culture (SD rats)	24 h	50 *μ*M CuCl_2_ combined with A*β* 50 *μ*M	↑ TNF-*α* and NO, ↑ iNOS	[126]
	BV2 cell line	24 h	0.01-5 *μ*M CuSO_4_ 0.01-5 *μ*M of A*β*	↓ Phagocytic activation of BV2 cells ↑ IL-1*β*, TNF-*α*, and IL-6	[127]

Zinc (Zn)	Primary microglia culture, C57BL6/J mouse	90 min	30 *μ*M ZnCl_2_	↑ Microglial activation. ↑ NF-*κ*B and NO production ↑ F4/80 expression	[133]
	Primary microglia culture C57BL6/J mouse. BV2 cell line	2 h	30-60 *μ*M ZnCl_2_	↑ iNOS mRNA	[134]

Cobalt (Co)	N9 cell line Primary microglia culture, Kunming mouse	24 h	1-500 *μ*M CoCl_2_	↑ NO, cytokines (TNF-*α* and IL-6) and chemokines ↑ iNOS mRNA	[135]
	Primary microglia culture C57BL6/J mouse. BV2 cell line	3, 6, 9, or 18 h	100 *μ*M CoCl_2_ stimulated with LPS. (0.25 *μ*g/mL)	↑ Induces hypoxia factor 1 (HIF1) ↓ NLRP3 ↓Caspase 1 and IL-1*β*	[136]
	Primary microglia culture (SD rats) BV2 cell line	24 h	250 *μ*M CoCl_2_	↑ HIF-1 and NF-*κ*B in rat microglial culture	[137]

Sprague-Dawley (SD) rats; ferroportin (FPN).

**Table 2:** Effects in microglia cells by nonessential metals.

Metal	Model	Time exposure	Concentration	Findings	Ref.
Lead (Pb)	Primary microglia culture (SD rats)	48 h	50 *μ*M Pb acetate (C_4_H_6_O_4_Pb)	↑ Microglia activation ↑ TNF-*α*, IL-1*β*, and iNOS	[148]
	C57BL6/J mouse (*in vivo*)	Daily for 3 days	Pb acetate (C_4_H_6_O_4_Pb, 15 mg/kg, i.p.)	↑ Microgliosis in the hippocampus *via* TLR4/MyD88/NF-*κ*B signaling cascades ↑ Expression of IL-1*β* and TNF-*α* ↑ p38-MAPK and ERK1/2	[152]
	C57BL6/J mouse (*in vivo*)	Exposed from PND 0 to PND 21	Pb (low dose), 30, and 430 ppm Pb acetate (C_4_H_6_O_4_Pb)	↓ Levels of C-C chemokine receptor type 7 (CCR7) ↓ Levels of MHCII	[153]
	BV-2 cell line	48 h	10 *μ*M Pb acetate (C_4_H_6_O_4_Pb)	↑ ROS and TNF-*α* levels significantly impacted the expression of 16 genes related to oxidative stress and antioxidant defenses in microglia	[154]

Aluminum (Al)	CB-84 (ATCC CRL-2467) murine microglial cells	8 h	2.0 *μ*M Al_2_(SO_4_)_3_	↓ TREM2 expression ↑ NF-*κ*B and miRNA-34a ↓ Phagocytic capacity ↑ Aggregation of A*β*42	[188]
	Male Wistar rats (*in vivo*)	Treated for 30 days Drinking water	Low-dose Al chloride (AlCl_3_) 10 ppm High-dose Al chloride (AlCl_3_) 100 ppm	↑ Lipid peroxidation (LPO) ↑ ROS formation ↑ Inflammatory response and microglial activation	[161]

Cadmium (Cd)	Primary microglia culture Fisher 344 rats	2, 6, or 24 h	0.062, 0.625, 1.25, or 2.50 *μ*M CdCl_2_	↑ Microglial activation ↑ ROS and the activation of transcription factors sensitive to redox like NF-*κ*B and AP-1	[165]
	C57BL6/N mice *in vivo* BV-2 cell line *in vitro*	2 weeks (i.p.) 24 h	5 mg/kg CdCl_2_ 1 *μ*g/mL CdCl_2_	↑ Levels of p- NF-*κ*B Cortex and hippocampus ↑ Iba-1, TNF-*α*, IL-1*β*, NOS2, ROS, LPO, p-NF-*κ*B, Bax, caspase 3, and PARP-1	[166]

Sprague-Dawley (SD) rats; intraperitoneal injection: i.p.

**Table 3:** Metals in Alzheimer's disease.

Metal	Study	Levels of metal	Findings	Ref.
*Essential*				
Manganese (Mn)	Patients and age-matched controls	Mn in blood, CDR (Controls) 0 = 11.20 ± 0.95 ng/ml. CDR 0.5 (mild cognitive impairment) = 12.37 ± 1.08 ng/ml. CDR 1 (mild dementia) = 9.63 ± 1.11 ng/ml. CDR > 2 (dementia) = 13.98 ± 0.88 ng/ml	Significant correlations of Mn with Mini-Mental State Examination score and Clinical Dementia Rating Scale score (CDR); plasma A*β* also increased with elevated Mn	[170]
Iron (Fe)	Study 37 participants aged between 62 and 89 years (22 cognitively normal, 15 MCI)	Levels of iron in the brain Controls = 1.16 ± 0.08 MCI = 1.5 ± 0.17	Confirmed the colocalization of brain Fe and A*β* plaques and promoted the development of the disease	[171]
Cooper (Cu)	Meta-analysis comparison between AD subjects and 200 controls	----	Confirmed higher levels of total Cu in AD subjects than in healthy controls (*p* < 0.0001)	[173]
	Frozen prefrontal brain tissues from patients with AD Braak stages V-VI	Control patients (*δ*65Cu = 0.60) AD brains (*δ*65Cu = 0.35)	Cu compositions of AD brains are statistically different compared to controls and correlate with Braak stages	[172]
Zinc (Zn)	Frozen prefrontal brain tissues from patients with AD Braak stages V-VI	Control patients (*δ*66 Zn = −0.6) AD brains (*δ*66 Zn = −0.4)	Zn of AD brains are statistically different compared to controls and correlate with Braak stages	[172]
	Nine AD subjects. Five controls	AD neutrophil = 51.4 ± 11.0 *μ*g/g Control neutrophil = 22.6 ± *μ*g/g	Zn levels are increased in senile plaque derived from patients diagnosed with AD	[123]
Cobalt (Co)	A 56-year-old woman with mental neuropathy	Co blood concentrations (>400 *μ*g/L; standard control: 0.18 ± 0.10 *μ*g/L). Co in the sural nerve was also elevated; Co (6.7 *μ*g/g vs. neuropathy controls <3.0 *μ*g/g)	Developed progressive sensory disturbance, hearing loss, and hypothyroidism. A sural nerve biopsy indicated axonopathy	[174]
	247 consecutive patients presented to an orthopedic clinic with an arthroprosthetic joint containing cobalt-chromium	Symptomatic patients with a blood Co level above 0.4 mcg/L or urine Co greater than 1 mcg/L underwent F-18 FDG PET brain imaging	All scanned patients had regions of significant hypometabolism. Neurological toxicity from elevated systemic Co	[175]

*Nonessential*				
Lead (Pb)	Case-control study, patients with AD	AD group = 22.22 + 28.57 mg/dL. Control group = 7.88 + 6.63 mg/dL	Pb levels were significantly higher in the patients with AD than in the controls	[176]
Aluminum (Al)	Human tissue was collected from deceased patients with AD	Al concentrations approach 12 *μ*g/g in some regions	Al levels have been traditionally linked to the pathogenesis of AD by its accumulation in the brain	[177]
	A 43-year-old man was exposed to high concentrations of Al	Al levels in the brain, especially the parietal and occipital lobes, were up to 5.58 and 4.45 *μ*g/g dry weight	The histology showed extensive and widespread hyperphosphorylated tau deposition in the neuritic plaques	[178]
	69-year-old man	Al content in each brain region varied from 0.45 (0.84) *μ*g/g dry wt. in the hippocampus to 1.75 (1.43) *μ*g/g dry wt. in the occipital lobe	Al content was high in occipital and parietal lobes and coincided with significant AD-related neuropathology	[180]
	12 donors diagnosed with familial AD	Al was found in all 144 tissues, and its concentration ranged from 0.01 to 35.65 *μ*g/g dry wt.	Supported by visual evidence of Al in brain tissue, it raises the possibility that genetic predisposition to AD is accompanied by a higher propensity to accumulate and retain Al in the brain	[179]
	A woman who is in 1998 had been exposed to very high and sustained levels of Al	----	Al was almost found intracellular in microglia, astrocytes, lymphocytes, and cells lining the choroid plexus	[181]
	Brain tissues	The Al content in the control (mean = 0.95) was significantly lower (*p* = 0.0006) than AD (mean = 1.69 *μ*g/g dry weight of tissue)	Al content of brain tissue in AD, autism spectrum disorder, and multiple sclerosis is significantly elevated	[182]
Cadmium (Cd)	Brain tissue (hippocampus and cerebral cortex) from AD and controls	Control hippocampus: 0.472. Control cortex: 0.496. AD hippocampus: 0.547. AD cortex: 0.518 *μ*g/g dry weight of tissue	Found that the AD brain had a higher concentration of Cd in the hippocampus and cerebral cortex	[184]
	*Post-mortem* frontal cortex samples from patients with AD	Control: 30 ng/g, AD: 20 ng/g	AD-related differences in metal levels with an elevation in Fe and a decrease in Cd	[185]
	Meta-analyses were used as the summary statistic for the difference in AD patients' toxic metals (Al, Hg, Cd, and Pb) compared to the controls	Circulatory Cd levels were significantly elevated in patients with AD (SMD = 0.62, 95% CI: 0.12, 1.11; *p* = 0.0144) compared to control subjects	Circulatory Cd levels were significantly elevated in patients with AD compared to control subjects	[186]

**Table 4:** Metals and Parkinson's disease.

Metal	Study	Levels of metal	Findings	Ref.
*Essential*				
Manganese (Mn)	Review of available clinical, neuroimaging, and neuropathological studies in humans and nonhuman primates exposed to Mn	----	Mn-induced Parkinsonism does not involve degeneration of midbrain dopamine neurons and that L DOPA is not an effective therapy	[189]
	Group 1 (G1): miners, welders, and bordering residents (they showed signs of Parkinsonism) Group 2 (G2): miners, welders, and bordering residents (had a routine clinical examination) Group 3 (G3): PD Group 4 (G4): cases of healthy and unexposed	The blood screening of manganese shows a high level upper than 15 *μ*g/L in the two first groups (G1 and G2)	High levels of manganese The authors underline the gravity of manganese-induced Parkinsonism	[190]
Iron (Fe)	Thirty-three PD patients and 26 age- and sex-matched healthy volunteers were included in this study	PD in SNc = 163.47 ± 49.16 ppb HV SNc = 85.18 ± 30.57 ppb *p* value < 0.01	PD is closely related to iron deposition in the SNc	[194]
Copper (Cu)	The brain tissue samples were from patients with idiopathic PD and incidental Lewy body disease (ILBD) and age-matched control subjects	Control subjects (SN) = 70 PD patients (SN) = 38 ILBD patients (SN) = 35 *μ*g/g dry weight	Decreased cellular Cu levels and disrupted Cu pathways in vulnerable brain regions in PD. Regional changes in SOD1 specific activity that reflect the pattern of neurodegeneration in PD	[196]
	50 PD patients diagnosed according to the UK PD Brain Bank criteria	Serum Cu Controls subjects = 1200 *μ*g/L PD subjects = 700 *μ*g/L	Low serum Cu concentration is related to PD development and predominantly affects the nonmotor symptoms of PD	[197]
Zinc (Zn)	Meta-analysis to evaluate whether circulating Zn levels in the serum, plasma, and cerebrospinal fluid (CSF) are altered in PD	Zn levels were significantly lower in PD patients vs. controls (SMD = −0.59; 95% CI [−1.06, −0.12]; *p* = 0.014)	This study suggests that reduced Zn levels in the serum and plasma are associated with an increased risk for PD	[199]
	60 patients who were registered in the 13th Regional Health Board (DIRES) and diagnosed with PD as determined by a certified specialty neurologist	PD patients with psychotic complications = 624.1 ± 56.9 *μ*g/g The patient group who did not report any psychotic complications = 513.9 ± 47.9 *μ*g/g Control group (459.3 ± 32.1 *μ*g/g)	Showed that patients with depression and patients with one or more of the psychotic complications of hallucination, illusion, paranoid ideation, altered dream phenomenon, and confusion exhibited significantly higher Zn concentrations in hair	[200]
	238 PD patients and 302 controls	Controls subjects = 1293 ± 385 *μ*g/L PD subjects = 923 ± 338 *μ*g/L	Zn level in PD patients was significantly decreased regardless of age status, suggesting that reduced plasma Zn concentration might be a potential signal for PD early warning	[201]
Cobalt (Co)	Two sites were selected: 1. Luqiao district, Taizhou 2. Huangyan District, Taizhou, as the reference area, 20 km north of Luqia	Blood concentrations Reference group = 0.35 ng/mL Exposed group = 0.5 ng/mL	Co in subjects' blood was associated with the alterations of the biomarkers of BBB and OS	[204]
	A 46-year-old man developed rapidly progressing Parkinson's disease symptoms after metal-on-metal total hip arthroplasty.	Serum Co: metal-on-metal total hip arthroplasty = 116 *μ*g/L Co	After revision, the patient's serum Co level fell below 1 *μ*g/L, and the PD symptoms improved	[203]
Lead (Pb)	Bone Pb concentrations were measured using 109 Cd excited K-shell X-ray fluorescence from 330 PD patients (216 men, 114 women) and 308 controls (172 men, 136 women)	OR for PD in the highest quartile was 3.21 [95% confidence interval (CI), 1.17–8.83]	Cumulative Pb exposure among typical PD patients seen in our movement disorders clinics strengthens the evidence that cumulative exposure to lead increases the risk of PD	[205]
Aluminum (Al)	Examined melanin-containing neurons of the substantia nigra in patients with PD and controls	PD 1 neuromelanin = 147.0 ± 7.0 Cytoplasm = 11.0 ± 2.4 Neutrophil = 9.8 ± 1.8 Control neuromelanin = 14.1 ± 1.4 Cytoplasm = 80.0 ± 1.0 Neutrophil = 4.5 ± 0.7	The accumulation of Al, which is known to promote oxidant stress, may account for the selective degeneration of neuromelanin-containing neurons in PD	[206]
	42 healthy controls and 45 drug naive PD patients	Control is 0.190 *μ*g/dL and 0.32 *μ*g/dL for PD	The serum Al level was significantly increased in PD patients	[208]
Cadmium (Cd)	A 64-year-old man suffered from acute exposure to cadmium	Cd concentration (blood 1.49 mg/dL, normal 0.11–0.66 mg/dL; urine 47.9 mg/L, normal 0.13–8.93 mg/L)	Three months after exposure, the patient developed Parkinsonian features. The case suggests that cadmium intoxication may damage the basal ganglia, resulting in Parkinsonism.	[212]
	Brain samples from people with neurodegenerative diseases	Cd was found in the locus coeruleus of all ten individuals examined	In individuals with AD or PD, a marked loss of locus coeruleus neurons was seen, with numerous collections of macrophage-bound and free neuromelanin pigment.	[211]

SN: substantia nigra; BBB: blood-brain barrier; OS: oxidative stress; PD: Parkinson's disease.
